RETRACTED

# Cluster-Based Immunotherapy for Patients with Recurrent Abortion Caused by Antiphospholipid Syndrome

**DOI:** 10.1155/2021/4581900

**Published:** 2021-09-18

**Authors:** Ruifang Wang, Juanjuan Yu, Zhen Yan, Xiaolin Cheng, Jian Chen, Yunhong Guo

**Affiliations:** The First Affiliated Hospital of Henan University of Science and Technology, Luoyang, Henan 471000, China

## Abstract

In order to diagnose patients with pregnancy and antiphospholipid antibody syndrome, provide early treatment, and effectively reduce the pregnancy outcome of the abnormal pregnancy, the effect of antiphospholipid syndrome (APS) immunotherapy on the incidence of abortion was discussed based on clustering algorithm. We selected 62 cases of APS leading to recurrent miscarriage patients, in the early pregnancy injection of low molecular heparin, intravenous drip proprocyclin, and oral tactics, using B-ultrasound images to observe the pregnancy ending. The results show that the hormone levels in the two groups were different before treatment (*P* > 0.05); after treatment, the HCG, E2, and P hormone levels in the two groups were significantly improved, and the HCG, E2, and P hormone levels in the observation group were significantly higher than those of the control group (*P* < 0.05); the abortion rate of patients in the observation group was significantly lower than that of the control group (*P* < 0.05); the antiphosphorus antibody of the study group was significantly higher than that of the control group. For APS patients, immunotherapy is effective. Antiphospholipid syndrome causes remarkable immunotherapy effect in patients with recurrent miscarriage, effectively improves the clinical symptoms of patients, improves antiprochemical antibody rosion, and improves the patient's pregnancy outcomes, which is worth promoting.

## 1. Introduction

With the rapid development of information technology, the data available are increasingly rich and the type of data is increasingly complex. Diet and housing are closely related to data analysis. Internet enterprises need a large number of data support service systems. On the other hand, traditional industries need to analyze past data to improve performance. Effective analysis of data has become one of the important factors in promoting social development. However, many times, massive, complex data make people dazzle. In the actual life, we can make a deep excavation of data by the clustering algorithm, making inductive reasoning, excavating potential patterns, understanding the profound impact of massive data, and changing our lives, work, and thinking [1]. Investigation of the effect of immunotherapy in patients with recurrent abortion caused by antiphospholipid syndrome (APS) was proposed. Ohams et al. proposed the theory of APS, explaining that this partially unexplained repeated abortion may be related to placental vascular thrombosis caused by immune imbalance [2]. Many patients have positive antiphospholipid antibodies, usually accompanied by infection symptoms due to immune imbalance, cervical secretions culture, group B streptococcus culture or mycoplasma chlamydia culture which are often positive, blood routine, and CRP abnormalities [3]. Cohen and BM believed that the positive rate of anticardiolipin antibody (ACL) was 30.0% in patients with recurrent abortion for 2 consecutive times and 32.5% in patients with recurrent abortion for ≥3 consecutive times. The current research cases are not enough, and further observation of the treatment effect of these patients can be carried out in the future to further make an accurate treatment analysis for these patients [4]. Before treatment, there was no significant difference in hormone levels between the two groups (*P* > 0.05). After treatment, the levels of HCG, E2, and P in 2 groups were significantly increased, and the levels of HCG, E2, and P in the observation group were significantly higher than those in the control group (*P* < 0.05). The abortion rate in the observation group was significantly lower than that in the control group (*P* < 0.05). The negative conversion rate of antiphospholipid antibody in the study group was significantly higher than that in the control group. Immunotherapy is effective in patients with APS. Clustering technology is an important research content in data mining, and people can use cluster analysis to group and classify, categorically, to better understand, research, and use data.

RETRACTED

## 2. Methods

### 2.1. B-Ultrasound Image Cluster

We use density-based clustering algorithms. In the space, the number of unit volumes is called the density of this point, intuitive, the same internal point is large, and the density of the class intervals is small. Based on density clustering according to the difference in spatial density, a point having a similar density is polygeneted into a class. DBSCAN is a typical density-based clustering algorithm that is a basic idea to connect adjacent high-density regions. For an object in the space, if the object is more than a given value MinPTS in the neighbor of a given radius *ε*, the object is referred to as a core point and otherwise referred to as a boundary object. All objects that can be reached by a core object constitute a class. Each object D in the image dataset is represented by a grayscale class, and the algorithm begins with an object D and extracts all the objects that are up from D density depending on parameter *ε* and minpts. If D is a core object, all objects from D can be recorded as the current class and is further expanded from them. If D is a boundary object, then D is recorded as a noise, and the algorithm extracts the next object for processing. The algorithm is in turn until a complete class is found. Then, a new start object is selected to start extension and the next class is obtained, until all objects are marked.

RETRACTED

### 2.2. Object and Grouping Method

A total of 120 patients with recurrent abortion caused by antiphospholipid syndrome from January 2018 to June 2019 were selected as the study subjects, and they were divided into the observation group (*n* = 60) and control group (*n* = 60) according to the random number table. By statistical analysis, the general data of the observation group and the control group were not significantly different (*P* > 0.05) and were comparable (Table 1).

Compared with the control group, ^*∗*^*P* < 0.05. It meets the diagnostic criteria of recurrent abortion caused by antiphospholipid syndrome. Patients with complete clinical data participated voluntarily and signed the informed consent. Patients with complicated hepatic and renal insufficiency or with other serious underlying diseases were excluded. The control group was treated with low-molecular-weight heparin and aspirin. The patients were given 100 mg aspirin orally once a day 4-5 months before pregnancy, subcutaneous injection of 0.4 ml low-molecular-weight heparin calcium once a day 2 months before pregnancy, and continued to use it for 32 weeks of gestation after pregnancy. During the treatment, the patient's blood flow and blood coagulation changes should be closely paid attention to, and the drug dosage should be adjusted according to the actual situation of the patient. The observation group received human immunoglobulin treatment on the basis of the control group: intravenous infusion of immunoglobulin C 5g, once a day, continuous use of 5 days in the first month, and continuous use of 3 days in the second and third months. Hormone level, antiphospholipid antibody negative turn, and abortion rate were observed and recorded in 2 groups. Data were expressed as (±*s*), the *t*-test was used for difference comparison, and the C2 test was used for counting data, *P* < 0.05.

### 2.3. Clinical Diagnosis and Treatment

Sixty-two APS-induced recurrent abortion patients from October 2014 to October 2016 with a history of more than three consecutive recurrent abortions were selected. They were 25 to 42 years old and tested positive for anticardiolipin antibody (ACA) twice. Chromosomal abnormalities of both husband and wife were excluded, and basic maternal diseases (thyroid dysfunction, reproductive system malformation, cervical insufficiency, and severe diabetes) were excluded. The gestational age of the patient's previous three abortions was 5 to 20 weeks. All the patients went to the doctor only after they were found to be pregnant this time, and the laboratory tests showed repeated positive ACA. From 5 to 7 weeks of pregnancy, they were given intravenous infusion of gamma globulin 5.0 g/d every month for continuous 5 days [5], low-molecular-weight heparin calcium 0.4 ml, twice a day, subcutaneously injected, and Seren 0.2 g, twice a day, orally. At the same time, if the symptoms of infection, such as vaginitis and abnormal blood routine and/or C-reactive protein (CRP), occurred, symptomatic treatment should be actively carried out, such as vaginal administration and intravenous injection of antibiotics. Patients need to go to the ophthalmology department to remove fundus lesions before application. Monthly review of coagulation function, blood routine, CRP, ACA, cervical secretions culture, cervical group B streptococcus examination, regular antenatal examination, and monitoring of fetal intrauterine conditions should be carried out [6].

RETRACTED

Among the 62 patients enrolled, 39 cases (62.9%) had pretermed delivery after 34 weeks of gestation, and 3 cases had preterm delivery due to premature rupture of membranes at 34 to 36 weeks of gestation. The other 36 cases were terminated at 37∼40 weeks of gestation, including 9 cases of vaginal delivery and 27 cases of cesarean section with “precious baby” as the indication. Apgar score of neonates after 34 weeks of gestation was 10 points, and there was no adverse pregnancy outcome. In addition, 6 cases of miscarriage occurred between 28 and 33 weeks of gestation, and 17 cases of miscarriage occurred between 10 and 26 weeks of gestation, as shown in Table 2.

In the clinical diagnosis and treatment, excluding the patient's own factors, about 50% of the patients with recurrent abortion etiology are unknown. Clinicians are often confused, and patients and families bear a lot of pain. The discovery of APS has raised hopes for the treatment of this subset of patients. It is a complex disease that seriously threatens the health of mothers and children. Its clinical manifestations mainly include thrombosis, recurrent abortion, intrauterine fetal death, preeclampsia, HELLP syndromes, FGR, and CAPS. APS is a noninflammatory autoimmune disease, clinically manifested by arterial and venous thrombosis, pathological pregnancy (early abortion and mid-late stillbirth), thrombocytopenia, and other symptoms. In patients with recurrent miscarriages, many patients have positive antiphospholipid antibodies, often accompanied by symptoms of infection due to immune imbalance, cervical secretions culture, group B *Streptococcus* culture or *Mycoplasma* chlamydia culture, and abnormal blood routine and CRP. Abortion in ACA-positive patients is mainly caused by thrombosis and inflammatory reactions in patients [7]. At present, there is still a lack of unified and standardized treatment for the treatment of parturient women with antiphospholipid antibody syndrome.

RETRACTED

## 3. Results and Analysis

For “symptomatic” B-ultrasound images, when the number of images is large and difficult to accurately diagnose the specific condition, clustering technology can be first used to divide the images into different groups, analyze each group of B-ultrasound images based on domain knowledge, and give the control group, so that the obtained image dataset can be used as a classified data source. By comparison of abortion rate and antiphospholipid antibody negative conversion rate between the 2 groups, the abortion rate of the observation group was significantly lower than that of the control group (*P* < 0.05). The antiphospholipid antibody negative conversion rate in the study group was significantly higher than that in the control group, and the difference was statistically significant (*P* < 0.05), as shown in Table 3.

Before treatment, there was no significant difference in hormone levels between the two groups (*P* > 0.05); after treatment, the levels of HCG, E2, and P hormones in the 2 groups were significantly increased, and the levels of HCG, E2, and P hormones in observation group were significantly higher than those in the control group (*P* < 0.05), as shown in Tables 4 and 5.

Antiphospholipid syndrome (APS) is an autoimmune disease caused by antiphospholipid antibodies, which is relatively common in clinic. If the pregnant patients with APS are not treated in time in the early stage, the probability of abortion is more than 50%, which seriously affects the physical and mental health of the patients, and the life safety of patients with serious conditions can be endangered. There are many clinical treatments for this disease, and most patients are still treated according to their clinical experience [8]. Studies have shown that immunotherapy can improve patients' clinical outcomes.

According to the characteristics of APS patients, the patients were given subcutaneous injection of low-molecular-weight heparin, intravenous drip of gamma globulin, and combined oral Xeneng treatment. The inhibitory effect of low-molecular-weight heparin on thrombosis and arteriovenous thrombosis in vivo and in vitro can stimulate endothelial cells to release tissue factor coagulation pathway inhibitors and activate protoplasmin, not neutralized by platelet factor 4, and has no significant impact on platelet function. It can be seen that heparin is a safe and effective anticoagulant. Previous studies have shown that heparin can improve microcirculation dysfunction. The effect on fetal placenta or fetal hypoxia is obvious. Hydroxychloroquine can reduce the production of AP1, which has the effect of antiplatelet aggregation and can inhibit the formation of placental thrombosis. Moreover, hydroxychloroquine is relatively safe for pregnant women and fetuses as the risk grade of pregnancy medication issued by the Food and Drug Administration of the United States is grade C. Intravenous dripping of gamma globulin is a kind of passive immunity, which can provide maternal immunity protection, reduce the risk of maternal infection, and reduce the occurrence of abortion induced by infection factors [9]. Experiments in China have shown that the application of gamma globulin can improve the success rate of pregnancy. Therefore, for patients with antiphospholipid antibody syndrome, immunotherapy combined with low-molecular-weight heparin, cyrenin, and gamma globulin is feasible and effective. However, in the treatment, there are many problems worth considering, such as the length of the combination of drugs; how to further adjust the dosage according to the inspection results; and duration of anti-infection medication and drug selection during pregnancy, for example, patients with combined functional insufficiency, whether cervical insufficiency is related to APS, and whether cervical ligation is needed. At present, there are clinical cases of APS screening and treatment before pregnancy [10]. Clinically, primary APS is more common, and such patients have immune abnormality before pregnancy, but it is often not until repeated early or middle pregnancy stillbirth or preeclampsia during pregnancy that patients pay enough attention to come to see a doctor.

RETRACTED

At present, the clinical treatment of recurrent abortion caused by antiphospholipid syndrome is mainly treated with aspirin, low-molecular-weight heparin, and other drugs, but the clinical effect is not satisfactory. Therefore, how to select reasonable and scientific treatment methods for recurrent abortion caused by antiphospholipid syndrome has become a clinical research hotspot [11]. Intravenous human immunoglobulin (HIMG) therapy is a new therapeutic method developed in recent years. The plasma of this treatment method is from a wide range of sources, mainly including autoantibodies, antiunique antibodies, and exogenous antibodies, which can give full play to the immunomodulatory effect of immunoglobulin C. At present, the mechanism of recurrent abortion caused by this immunotherapy in the treatment of antiphospholipid syndrome is still not clear, mainly including immunoglobulin C which can effectively inhibit T cells or NK cells and reduce pathological immune response. It can competitively inhibit multiple antibody receptors on idiotypic response sites. It can effectively inhibit complement binding and activation, regulating cytokine production and so on. The results of this study showed that, before treatment, there was no statistical significance in hormone levels between the 2 groups (*P* > 0.05). After treatment, the levels of HCG, E2, and P in the 2 groups were significantly increased, and the levels of HCG, E2, and P in the observation group were significantly higher than those in the control group (*P* < 0.05). The abortion rate in the observation group was significantly lower than that in the control group (*P* < 0.05). The negative conversion rate of antiphospholipid antibody in the study group was significantly higher than that in the control group (*P* < 0.05), further indicating that immunotherapy has a significant effect on patients with recurrent abortion caused by antiphospholipid syndrome [12].

## 4. Conclusions

This paper proposes an immunotherapeutic effect to discuss antiphospholipid syndrome (APS) causing abortion patients. Before treatment, there was no significant difference in hormone levels in the two groups (*P* > 0.05); after treatment, HCG, E2, and *p* hormone levels in two groups were significantly improved, and HCG, E2, and *p* housing levels in the observation group were significantly higher than that of the control group (*P* < 0.05); the abortion rate of patients in the observation group was significantly lower than that of the control group (*P* < 0.05); the antiphosphorus antibody of the study group was significantly higher than that of the control group. Traditional clustering or module optimization drawing methods typically only assign a vertex of the figure to a unique cluster. However, in some cases, there is an inevitable overlap factor between clusters and clusters of the figure. The detection of overlapping clusters in the figure began to become one of the research hotspots of current graph clusters. Antiphospholipid syndrome causes remarkable immunotherapy effect in patients with recurrent miscarriage, effectively improves the clinical symptoms of patients, improves antiprochemical antibody rosion, and improves the patient's pregnancy outcomes, which is worth promoting.

## Figures and Tables

**Table 1:** Clinical data analysis of the two groups of patients.

Group	Age	Frequency of natural flow
Observation group (*n* = 60)	27.2 ± 4.5	3.21 ± 1.42
The control group (*n* = 60)	26.8 ± 4.4	3.29 ± 1.38

RETRACTED

**Table 2:** Data of childbirth in the pregnancy cycle.

The pregnancy period	Preterm birth	Vaginal delivery	Missed abortion	Spontaneous abortion	Cesarean delivery
34∼36 weeks	3	0	0	0	0
37∼40 weeks	0	9	0	0	27
28∼33 weeks	0	0	0	0	6
10∼26 weeks	0	0	9	8	0

**Table 3:** Comparison of abortion rate and antiphospholipid antibody negative conversion rate between the two groups.

Group	Abortion rate	Negative conversion rate of antiphospholipid antibodies
Observation group	14 (23.33)	57 (95)
The control group	27 (45)	43 (71.67)
*x* ^2^	4.294	4.025
*P* value	<0.05	<0.05

**Table 4:** Comparison of hormone levels between the two groups.

Group	Before the treatment	After treatment
Observation group	997.38 ± 102.44	6724.25 ± 593.30
The control group	999.27 ± 104.23	6103.25 ± 4983.71
T	1.093	4.298
*P* value	>0.05	<0.05

**Table 5:** Comparison of hormone levels between the two groups.

Group	Before the treatment	After treatment	Before the treatment	After treatment
Observation group	365.38 ± 36.54	462.95 ± 36.58	8.14 ± 2.11	27.42 ± 4.28
The control group	363.29 ± 40.15	410.26 ± 42.18	8.29 ± 2.31	21.03 ± 4.93
T	0.027	6.024	0.024	6.039
*P* value	>0.05	<0.05	>0.05	<0.05

## Data Availability

The data used to support the findings of this study are available from the corresponding author upon request.
